The article "Concordane of OSTA and lumbar spine BMD by DXA in identifying risk of osteoporosis" was published in 2006. Journal: J Orthop Surg Res.

# Concordane of OSTA and lumbar spine BMD by DXA in identifying risk of osteoporosis

**DOI:** 10.1186/1749-799X-1-14

**Published:** 2006-11-21

**Authors:** ChunYan Lu, DeCai Chen, YunHua Cai, SongQuan Wei

**Affiliations:** 1 Department of Endocrinology, West China hospital of SiChuan University, ChengDu, China; 2 Department of Endocrinology, County hospital of QianWei, SiChuan, China

## Abstract

**Objective:**

To investigate the accuracy of Osteoporosis Self-assessment Tool for Asians (OSTA) in identifying the risk of osteoporosis in postmenopausal women. To validate use of OSTA risk index by comparing it with the bone mineral density (BMD) of lumbar spine measured by dual energy X-ray absorptiometry (DXA).

**Methods:**

The data of lumbar spine BMD (LS BMD) measurements by DXA of 218 postmenopausal women of Han nationality in Sichuan province were compared with OSTA risk index. The concordance of OSTA and LS BMD were calculated and analyzed by fourfold table and receiver operating characteristic (ROC) curve.

**Results:**

The prevalence of osteoporosis in these women was 40.4% and 61.5%, with the LS BMD T score cutoffs -2.5 and -2.0, respectively. The sensitivity, specificity, and accuracy of OSTA risk index compared with T score cutoff -2.5 of LS BMD were 59.1%, 56.9% and 57.8%, respectively, while they were 57.5%, 63.1%, 59.6% by T score cutoff -2.0.

**Conclusion:**

For identifying risk of osteoporosis, the concurrence was lower than those reported studies when comparing LS BMD measurements to OSTA risk index in Chinese Han nationality postmenopausal women of Sichuan province. Physicians should identify women who need BMD measurement according to more factors rather than age and body weight.

## 1. Background

According to the improvement of living standard and life expectancy, osteoporosis (OP) is becoming one of the most common pubic healthy problems in China and worldwide. The prevalence of osteoporosis is progressively increasing. The most severe complication of OP is fracture, which brings great burden to individual, family and society.

Osteoporosis is very common among postmenopausal women [1-3], while women of high risk are often asymptomatic. Therefore, early screening and evaluation of osteoporosis in postmenopausal women are important. It is widely accepted that bone mineral density (BMD) measurement measured by dual X-ray absorptiometry (DXA) is the golden standard of diagnosis of OP. Because of the limited availability and rather expensive cost of DXA, simple tools in identifying women needed DXA measurements have developed.

The Osteoporosis Self-assessment Tool for Asians (OSTA) is an index using chart or formula to predict low BMD simply on the basis of age and weight[4]. It was firstly proposed by Koh LK, which had a sensitivity of 91% and specificity of 45% in identifying women of high risk when compared with final results of femoral neck BMD measurement in Asia women. The index of Osteoporosis Self-assessment Tool (OST) is calculated by the same formula or chart of OSTA, which is reported to predict low BMD in other races of people using different cutoff values[5].

The article "Concordane of OSTA and lumbar spine BMD by DXA in identifying risk of osteoporosis" was published in 2006. Journal: J Orthop Surg Res.

In this article, 218 Chinese women of Han nationality in Sichuan province were assessed by OSTA index and the usefulness of OSTA was evaluated to predict osteoporosis in comparing with LS BMD which measured by DXA.

## 2. Data and methods

This study is a diagnostic test. We analyzed the database of DXA measurement for lumbar spine BMD (LS BMD) from August 1^st ^2005 to September 30^th ^2005 in our hospital. Most of the patients did not measure femoral neck or hip BMD. In-patient and out-patient postmenopausal women of Han nationality from Sichuan province were selected for further evaluation, among which enrolled in a physical examination clinic, rehabilitation department, geriatric department and endocrinology department were recruited. Patients were ineligible if they had a history in their case files of advanced osteoarthritis, hyperthyroidism, hyperparathyroidism, renal failure, and other knowing severe diseases or conditions that could interfere with bone metabolism. Finally, 218 postmenopausal women were eligible and applied the OSTA index.

LS BMD by DXA was measured with Challenger densitometer (DMS, France), which uses the DMS reference source for the spine. A spine phantom was measured every week to keep the precision error less than 2%. All measurements were completed by one operator. T scores of lumbar spine L_2 _to L_4 _were obtained and osteoporosis was defined as T scores of any site equal to or less than -2.5[6]. In addition, when compared with the OSTA index, a T score cutoff for osteoporosis of -2.0 were also applied, according to the consensus of some specialists in China[7]. These postmenopausal women were identified at various BMD thresholds (T score values of -2.0 and -2.5) for osteoporosis and non-osteoporosis (osteopenia or normal).

OSTA index was derived according to the formula of 0.2 × (weight in kilograms – age in years), truncated to an integer[4,5,8]. Three risk categories were used for the index according to its developer's recommendations[4] and in our study, dichotomous cutoff for Asian women were used as the following: ≥ 0 for low risk and < 0 for moderate-high risk.

A fourfold table was applied to calculate the sensitivity (sen.), specificity (spe.), and accuracy of OSTA compared with different T score cutoffs of LS BMD by DXA. Receiver operating characteristic curves (ROC curves) were constructed and the areas under curve (AUC) as well as its 95% confidence interval (95% CI) was estimated by using SPSS statistical software10.0 (SPSS Inc.). The prevalence of osteoporosis was examined across different categories of the OSTA risk index.

The article "Concordane of OSTA and lumbar spine BMD by DXA in identifying risk of osteoporosis" was published in 2006. Journal: J Orthop Surg Res.

## 3. Results

The mean age of the postmenopausal women in this study was 59.0 ± 9.2 years, and the mean weight was 56.7 ± 9.8 kg. The prevalence of osteoporosis at lumbar spine increased progressively with age (Figure 1). Of all the women in our sample, 40.4% (T ≤ -2.5) and 61.5% (T ≤ -2.0) were osteoporotic at L_2–4_, respectively. The OSTA index varied between -9 to 6, and the percent distribution of the women according to the OSTA index is shown in Figure 2. On the basis of categories used in Asian women[4], there are 50.5% women (n = 110) of low risk, 42.2% (n = 92) of moderate risk, and 7.3% (n = 16) of high risk, respectively. Figure 3 shows the different cutoffs for LS BMD T score by DXA and the categories of low, moderate, and high risk of osteoporosis by OSTA index.

**Figure 1:** Prevalence of osteoporosis by age and T score cutoffs (T ≤ -2.5 and T ≤ -2.0) of DXA measurement.

**Figure 2:** Distribution of the patients according to their OSTA risk index.

**Figure 3:** Prevalence of osteoporosis according to various T score cutoffs at different levels of OSTA risk index. (Categorization used in Asian women by koh et al[4]. Numbers of women in low, moderate, and high risk group are 110, 92, 16, respectively.)

Table 1 was the fourfold table of OSTA in assessing risk of osteoporosis comparing with LS BMD according to various cutoffs. Performance of OSTA risk index comparing with LS BMD by DXA and T score cutoffs was shown in table 2. The results showed that the sensitivity, specificity, and accuracy were 59.1%, 56.9%, 57.8% (LS BMD T score cutoff -2.5), and 57.5%, 63.1%, 59.6%(LS BMD T score cutoff -2.0), respectively. The OSTA yielded AUC of 0.615 (95% CI 0.537 to 0.692) and 0.628 (95% CI 0.553 to 0.703) for LS BMD by DXA T score of -2.5 or less and -2.0 or less, respectively (Figure 4 and 5).

**Table 1:** Fourfold table of OSTA comparing with LS BMD by DXA

	LS BMD by DXA					
	
	T ≤ -2.5			T ≤ -2.0		
OSTA index	OP	non-OP	total	OP	non-OP	total
moderate-high risk	52	56	108	77	31	108
low risk	36	74	110	57	53	110
total	88	130	218	134	84	218

**Table 2:** Performance of OSTA index by LS BMD and various T score cutoffs

	Sen.	Spe.	Accuracy
T ≤ -2.5	59.1%	56.9%	57.8%
T ≤ -2.0	57.5%	63.1%	59.6%

**Figure 4:** The ROC curve for OSTA index using LS BMD T score cutoff -2.5 by DXA measurement.

The article "Concordane of OSTA and lumbar spine BMD by DXA in identifying risk of osteoporosis" was published in 2006. Journal: J Orthop Surg Res.

**Figure 5:** The ROC curve for OSTA index using LS BMD T score cutoff -2.0 by DXA measurement.

## 4. Discussion

It's never ending for specialists to find out an easy tool for osteoporosis risk evaluation. The Chinese Medical Association recommended that all women aged 65 and older or postmenopausal women with one or more risk factors should have BMD measurements[9]. But it is not possible for all women satisfied with the conditions mentioned above to receive DXA measurements in China, because of little physicians' and patients' awareness, little public heath policy support, and so on. Therefore, we want to find out patients in high risk of osteoporosis using simple tools such as OSTA, which had been validated well in classifying the osteoporotic risk among postmenopausal women.

There are many risk assessment indices in identifying women at moderate or high risk of osteoporosis who need BMD measurements by DXA, such as Osteoporosis Index of Risk (OSIRIS), Simple Calculated Osteoporosis Risk Estimation (SCORE), Osteoporosis Risk Assessment Instrument (ORAI), and OSTA. All of these tools were predicting osteoporosis risk according to age, weight, race, history of fracture, history of medication, and so on. The main results were displayed in table 3. It was said the OSTA, based only on age and weight, could perform well in assessing risk categories[4,5,8,10-14]. In our study involving 218 Asian postmenopausal women of Han nationality in Sichuan Province with a mean age of 59.0 years, the OSTA index did not perform very well in identifying women of high risk whose LS BMD by DXA measurements were very low (T score less than -2.5 or -2.0). For example, among the 88 (40.4%) women of osteoporosis using a T score cutoff -2.5 by DXA, only 52 women were identified moderate or high risk by OSTA risk index. It means 41% women of osteoporosis will be neglected if they were assessed only by OSTA index. Meanwhile, among the 130 women of non-OP (osteopenia or normal bone mass), only 74 (57%) women were low risk by OSTA who did not need BMD measurement.

**Table 3:** Results of OST(A) in diagnostic studies.

Investigator	Publication time	Race	Sample size	Sen.	Spe.
Koh LK^(4)^	2001	Asian women	860	91%	45%
Kung AW^(10)^	2003	Hong Kong women	722	79–88%	54–60%
Park HM^(11)^	2003	Korea women	1101	80–87%	67–72%
Yang NP^(12)^	2004	Taiwan women	3456	Compared with QUS*	
Wallace LS^(13)^	2004	African-American women	174	83.61%	53.85%
Cadarette SM^(14)^	2004	Canadian white women	190	> 90%	40%
Richy F^(5)^	2004	Belgian Caucasian women	4035	85%	37%
Adler RA^(8)^	2003	American white men	181	93%	66%

* QUS means Calcaneal quantitative ultrasound.

We found the performance of OSTA risk index is not as satisfied as those reported in Asian or other races and it can not help us precisely to give judgement on whether a DXA measurement of LS BMD should be given to a postmenopausal women or not. Because our subjects were from hospital, not from an epidemiologic investigation, the prevalence of osteoporosis was rather higher than those reported in Asian women[4]. Through a woman's life, there are so many risk factors for osteoporosis, such as age, race, hormone conditions, heredity, weight, nutritional status, history of fracture, childbearing, and so on[15]. We think there were limitations in OSTA risk index by using only age and weight. According to the OSTA formula, if the weight (in kilograms) of a woman surpasses her age (in years), she will always be in low risk of osteoporosis. It is of some absurd for you to tell your patient that when she was 90 years old, she should keep the body weight 90 kg for prevention of osteoporosis.

The article "Concordane of OSTA and lumbar spine BMD by DXA in identifying risk of osteoporosis" was published in 2006. Journal: J Orthop Surg Res.

The identification of low bone mass in postmenopausal women should be emphasized because of the severe complications. Although some experts should give advice to their patients, most physicians and patients in our country are not aware of osteoporosis. It is only appropriately diagnosed and treated in a very small proportion of patients, even if they had a prior history of osteoporotic fracture. Up to now, BMD measurement is still the golden standard of osteoporosis diagnosis. We recommended that physicians should identify women who are likely to have low BMD according to much more factors than OSTA risk index.

The limitation of this study is that not all patients measured femoral neck BMD, so the data did not compared with OSTA index. Although BMD measurements of total hip and femoral neck were easily influenced by body position, they could be alternative sites for identifying osteoporosis, especially when false high lumbar spine BMD were found because of vertebral fractures, hyperostosis, aortic calcification, and so on.

## 5. Conclusion

A risk index of osteoporosis like OSTA has its characteristic of calculating simply and quickly. But the validation of its use in our hospital for postmenopausal women who underwent LS BMD measurements by DXA was somewhat disappointed. The OSTA risk index may not be a very good method in identifying postmenopausal women at high risk of osteoporosis, as measured by DXA, in Sichuan province.
